# Differential inductions of phenylalanine ammonia-lyase and chalcone synthase during wounding, salicylic acid treatment, and salinity stress in safflower, *Carthamus tinctorius*

**DOI:** 10.1042/BSR20140026

**Published:** 2014-06-25

**Authors:** Sara Dehghan, Mahnaz Sadeghi, Anne Pöppel, Rainer Fischer, Reinhard Lakes-Harlan, Hamid Reza Kavousi, Andreas Vilcinskas, Mohammad Rahnamaeian

**Affiliations:** *Department of Plant Biotechnology, College of Agriculture, Shahid Bahonar University of Kerman, P. O. Box: 76169-133, Kerman, Iran; †LOEWE Center for Insect Biotechnology and Bioresources, Fraunhofer Institute for Molecular Biology and Applied Ecology (IME), Giessen, Winchesterstrasse 2, 35394, Giessen, Germany; ‡Interdisciplinary Research Center, Institute for Phytopathology and Applied Zoology, Justus Liebig University of Giessen, Heinrich-Buff-Ring 26-32, 35392, Giessen, Germany; §AG Integrative Sensory Physiology, Institute for Animal Physiology, Justus Liebig University of Giessen, Heinrich-Buff-Ring 26, 35392, Giessen, Germany

**Keywords:** defence response, safflower, salicylic acid (SA), salinity, semi-quantitative RT–PCR, wounding, 4CL, 4-Coumarate:CoA ligase, aa, amino acid, C4H, cinnamate 4-hydroxylase, CHS, chalcone synthase, hat, hours after treatment, PAL, phenylalanine ammonia-lyase, SA, salicylic acid

## Abstract

Safflower (*Carthamus tinctorius* L.) serves as a reference dicot for investigation of defence mechanisms in Asteraceae due to abundant secondary metabolites and high resistance/tolerance to environmental stresses. In plants, phenylpropanoid and flavonoid pathways are considered as two central defence signalling cascades in stress conditions. Here, we describe the isolation of two major genes in these pathways, *Ct*PAL (phenylalanine ammonia-lyase) and *Ct*CHS (chalcone synthase) in safflower along with monitoring their expression profiles in different stress circumstances. The aa (amino acid) sequence of isolated region of *Ct*PAL possesses the maximum identity up to 96% to its orthologue in *Cynara scolymus*, while that of *Ct*CHS retains the highest identity to its orthologue in *Callistephus chinensis* up to 96%. Experiments for gene expression profiling of *Ct*PAL and *Ct*CHS were performed after the treatment of seedlings with 0.1 and 1 mM SA (salicylic acid), wounding and salinity stress. The results of semi-quantitative RT–PCR revealed that both *Ct*PAL and *Ct*CHS genes are further responsive to higher concentration of SA with dissimilar patterns. Regarding wounding stress, *Ct*PAL gets slightly induced upon injury at 3 hat (hours after treatment) (hat), whereas *Ct*CHS gets greatly induced at 3 hat and levels off gradually afterward. Upon salinity stress, CtPAL displays a similar expression pattern by getting slightly induced at 3 hat, but *Ct*CHS exhibits a biphasic expression profile with two prominent peaks at 3 and 24 hat. These results substantiate the involvement of phenylpropanoid and particularly flavonoid pathways in safflower during wounding and especially salinity stress.

## INTRODUCTION

As ground-anchored sessile organisms, plants have evolved diverse adaptive and defence mechanisms in order to survive in threatening environmental conditions. Growth-limiting factors including drought, salinity, cold, UV rays as well as pathogenic micro-organisms, e.g. fungi, bacteria, viruses, etc. all can jeopardize the plant life if not negated by plant protective responses. In breeding programmes, identification of protecting factors in plants against challenging factors is a prerequisite. In this context, keeping our efforts in identification and characterization of involved genes in plant responses to biotic and abiotic stresses [1–4], we report in this study the isolation as well as functional characterization of two genes in phenylpropanoid and flavonoid pathways, i.e. PAL (phenylalanine ammonia-lyase) and CHS (chalcone synthase) in safflower (*Carthamus tinctorius*) during salinity stress, wounding and SA (salicylic acid) treatment as an inducer of acquired resistance and PR genes expression [5].

We have been recently working on safflower [4] given that this industrial medicinal oil-seed plant has a rich germplasm collection in Iran and shows high levels of tolerance/resistance to environmental stresses. Safflower is a long-day, herbaceous, annual, self-compatible member of Asteraceae family and *Carthamus* genus. Having a well-developed root system, safflower is an ideal plant in arid and semi-arid climates [6,7]. Iran is one of the richest countries regarding safflower germplasms including domestic and wild species [8]. A variety of abiotic/biotic stresses challenges the safflower namely high-temperature, high relative humidity, long rainfalls, drought, cold and salinity as well as many fungal and a few bacterial and viral pathogens [9]. However, owing to high tolerance/resistance of safflower to environmental stresses, this plant might be considered as a reference plant for studying the defence mechanisms. Plant responses to environmental stimuli are governed by a complicated multi-player crosstalk among different defence pathways. In higher plants, phenylpropanoid biosynthetic pathway produces the important metabolites, e.g. flavonoids, isoflavonoids, lignin, anthocyanin, phytoalexins, antimicrobial furanocoumarins, hydroxyl cinnamate esters and phenolic esters, which are all critical players in development, structural protection, defence responses to microbial attacks and tolerance to abiotic stimuli [10,11]. As phenylpropanoid pathway is a gateway for production of many secondary metabolites [12,13], the investigation of characteristics as well as expression patterns of involved genes in production of these metabolites, e.g. PAL and CHS, for a better understanding of defence mechanisms towards various stresses appears significantly useful. PAL is the initial enzyme in phenylpropanoid pathway and the key participant in the lignification process [12], which converts the phenylalanine to trans-cinnamic acid via non-oxidative removal of ammonia as depicted in Figure 1. PAL is a critical enzyme for plant responses to environmental stresses as if its *de novo* synthesis is activated following pathogen attack, wounding, UV irradiation, as well as iron and phosphate depletion [19]. It is, also, responsive to phytohormones ethylene, jasmonic acid, SA and methyl jasmonate [20–24]. CHS is another important enzyme in phenylpropanoid cascade and the key enzyme in flavonoid biosynthesis (Figure 1). Flavonoids are the major groups of plant secondary metabolites with essential roles in physiological processes. Flavonoids have not only been considered for their significance in plants nutritional value [25], but are also important in terms of plant protection against UV rays, pathogen attacks and herbivores [26–29].

**Figure 1:** Phenylpropanoid and flavonoid pathways in plants PAL and CHS in respective phenylpropanoid and flavonoid pathways are shown in red. The scheme was adapted after [14–18].

Since only one gene, i.e. C4H (cinnamate 4-hydroxylase), of phenylpropanoid pathway in safflower has been isolated and characterized so far [4], in this study the coding sequences of safflower PAL (*Ct*PAL) and CHS (*Ct*CHS), which are typically encoded by small multi-gene families, have been partially isolated and their expression profiles during SA treatment, wounding and salinity stress were monitored in order to further dissect the high levels of resistance/tolerance of safflower to different environmental stresses.

## MATERIALS AND METHODS

### Plant material and growth condition

Seeds of safflower var. 22-191 (kindly provided by Dr Mahammadinejad, Department of Agronomy, Shahid Bahonar University of Kerman, Iran) were sterilized with 70% (v/v) ethanol and sodium hypochlorite [5% (w/v) active chlorine] for 2 and 15 min, respectively. Having vernalized at 4°C for 2 h, seeds were sown on water-soaked sterile filter papers. The germinated seeds were transplanted into 15-cm-diameter pots filled with prewashed sand and kept in the greenhouse at 26±2°C and photoperiod of 16 h with every other 2 days irrigation regime. Fertilization by Hoagland solution was performed once a week.

### Isolation of partial sequences of *Ct*PAL and *Ct*CHS genes

Isolation of genomic DNA from leaves was carried out after Saghai-Maroof et al. [30]. The available coding sequences of PAL orthologues in members of Asteraceae family, i.e. *Helianthus annuus*, *Rudbeckia hirta*, *Cynara scolymus* and *Gynara bicolor*, were used to design the isolating primer pair for *Ct*PAL. Likewise, the coding sequences of CHS genes in *R. hirta*, *Lactuca sativa*, *G. bicolor* and *Silybum marianum* were considered to design the isolating primers for *Ct*CHS. Table 1 shows the sequences of primers used in this study, which were synthesized by Eurofin MWG Operon (Germany). Amplicons of *Ct*PAL (872 bp) and *Ct*CHS (559 bp) were obtained by performing PCR on genomic DNA using 1 pmol of gene-specific primer pairs. Temperatures of annealing for *Ct*PAL and *Ct*CHS were 51 and 56°C, respectively.

**Table 1:** Sequences of primer pairs used for isolation and semi-quantitative RT–PCR in this study

Gene	Primer	Sequence (5′-3′)	Amplicon size (bp)
Phenylalanine ammonia-lyase (isolation)	*Ct*-PAL-Fwd	CTCCTCCAGGGTTACTCC	872
	*Ct*-PAL-Rev	CCTTTGAACCCGTAATCC	
Chalcone synthase (isolation; RT–PCR)	*Ct*-CHS-Fwd	AAACGCTTCATGATGTACCA	559
	*Ct*-CHS-Rev	GCCGACTTCTTCCTCATCTC	
Phenylalanine ammonia-lyase (RT–PCR)	*Ct*-PAL2-Fwd	GCAGAAACCCAAACAAGA	267
	*Ct-*PAL2-Rev	TTAACAAGCTCGGAGAATT	
18S rRNA (RT–PCR)	18S rRNA-Fwd	ACTCACCTCAAGACT	199
	18S rRNA-Rev	CTTTGGCACATCC	

### Cloning of *Ct*PAL and *Ct*CHS amplicons into sequencing vector

To clone the amplicons of *Ct*PAL and *Ct*CHS into pTZ57R/T vector, InsTAclone™ PCR Cloning Kit (Thermo SCIENTIFIC, # K1213) and competent cells of *Escherichia coli* strain JM107 were recruited. In brief, based upon blue/white screening, recombinant colonies were selected for DNA extraction by GF-1 Plasmid DNA Extraction Kit (Vivantis). Sequences of isolated region of *Ct*PAL and *Ct*CHS genes were obtained using M13 universal primers (Faza Pajooh Biotech). Sequences were certified by means of Chromas Lite 2.01 (Technelysium) after clipping the vector sequence.

### Conserved domains, homology and phylogenetic analyses

Bioinformatics analysis of *Ct*PAL and *Ct*CHS aa (amino acid) sequences were performed in conserved domain platform [31,32] at http://www.ncbi.nlm.nih.gov/Structure/cdd/cdd.shtml. The aa sequences of *Ct*PAL and *Ct*CHS were analysed for homology using ClustalW [33]. Constructions of phylogenetic tree based on nucleotide sequence for *Ct*PAL and *Ct*CHS genes were carried out using Phylogeny.fr program [34–36]. Briefly, sequences were aligned with the highest accuracy by MUSCLE [37]. Phylogenetic trees were constructed based upon the maximum likelihood approach executed in PhyML 3.0 software [38,39]. Graphical demonstration of trees was completed by TreeDyn [40].

### Gene expression analyses

Wounding, salinity and SA treatments were all performed on 14-day-old seedlings. For wounding, leaves were comparably equally pressed with sterile blunt-nosed thumb forceps. For salinity, seedlings were drenched with 150 mM sodium chloride solution. For SA treatment, two experimental groups of 0.1 and 1 mM SA were considered. SA solutions were applied on leaves using sprayer. Following each treatment, samplings were done in a time course, i.e. 0, 3, 6, 12, 24 and 48 hat (hours after treatment). Taken into account the potential diurnal rhythm in the gene expression patterns, all treatments were started at 8 am.

### RNA extraction and cDNA synthesis

RNAs were extracted by means of RNX™ Plus Kit (Cinnagen) from the treated seedlings according to manufacturer's instructions. Next to DNaseI treatment of RNA samples, 1 μg of RNAs, using RevertAid First Strand cDNA Synthesis Kit (Thermo SCIENTIFIC, # K1691), was reverse transcribed to corresponding cDNAs, which were later used as templates for semi-quantitative RT–PCR.

### Semi-quantitative RT–PCR

To normalize the cDNA amounts of different time points in each treatment, we considered the PCR product intensity of 18S rRNA as the house-keeping gene. The primer pairs for *Ct*PAL and *Ct*CHS are given in Table 1. The PCR thermal profile was: 98°C (5 min) followed by 35 cycles of 98°C (10 s), 52°C (15 s) and 72°C (1 min), and a final extension time at 72°C for 10 min. An independent experiment was carried out to verify the linear amplification in such setting. The interpretation was based on the intensity of PCR products, corresponding to gene transcription levels.

## RESULTS AND DISCUSSION

In this study, besides the partial isolation of coding sequences of PAL (*Ct*PAL) and CHS (*Ct*CHS) in safflower, the consequences of salinity stress, wounding, as well as SA treatment, as an stimulus of plant defence against pathogen attacks, on expression profiles of these genes were investigated. Very little information, at the molecular level, is available in safflower, thereby keeping our work on safflower [4], we focused, in this study, on *Ct*PAL and *Ct*CHS genes, two critical genes in phenylpropanoid and flavonoid pathways (Figure 1). These pathways have been proved to be highly critical in plant protective reactions during biotic and abiotic stresses [2].

### Conserved domains, homology and phylogenetic analyses of *Ct*PAL

According to the results of conserved domain analysis, the isolated region of safflower PAL, *Ct*PAL, contains the conserved domain of Lyase class I_like superfamily (cl00013) accommodating HAL (histidine ammonia-lyase) and PAL. PAL–HAL conserved domain (cd00332) is present in plants, fungi, several bacteria and animals [41]. Phenylalanine and HALs, which are active as homotetramers [42], catalyse the beta-elimination of ammonia from respective phenylalanine and histidine [43]. Like other homotetrameric enzymes in this family, safflower PAL possesses four active sites, as detected in conserved domain platform. PAL, present in plants and fungi, catalyses the conversion of L-phenylalanine to E-cinnamic acid. The aa sequence of the isolated *Ct*PAL fragment comprising 291 aa (GenBank: AFK25796) was used as an initial query to search, using the protein–protein BLAST tool, against the non-redundant protein sequences. As a result, the isolated region of *Ct*PAL shows the maximum identity up to 96% to PAL of *C. scolymus*, followed by lettuce PAL (*L. sativa*) up to 95%, *G. bicolor* and *R. hirta* up to 94% and sunflower PAL (*H. annuus*) and *Ageratina adenophora* up to 92%, which are all in Asteraceae family as shown in Figure 2(A). The inferred evolutionary history of PAL nucleotide sequences from several plant species and the corresponding phylogenetic tree bring to light a rather conserved PAL orthologues in Asterids with low genetic distance (0.2) as depicted in Figure 2(B). The coding sequence of *Ct*PAL was deposited in GenBank under the accession number JN998609.

**Figure 2:** Amino acid sequence alignment (A) and phylogenetic analysis (B) of CtPAL orthologues Sequence alignment and aa conservation profile for PAL orthologues were generated by ClustalW. Constructions of phylogenetic tree based on nucleotide sequence for PAL gene was carried out by Phylogeny.fr program. In brief, sequences were aligned with the highest accuracy by MUSCLE. Phylogenetic tree was constructed based upon the maximum likelihood approach executed in PhyML 3.0 software. Graphical demonstration of tree was completed by TreeDyn. Accession numbers for (A): *Carthamus tinctorius* (AFK25796); *Cynara cardunculus* (CAL91171); *Lactuca sativa* (AAL55242); *Chrysanthemum boreale* (AGU91428); *Rudbeckia hirta* (ABN79671); *Gynura bicolor* (BAJ17655); *Helianthus annuus* (CAA73065); *Ageratina adenophora* (ACT53399); *Platycodon grandiflorus* (AEM63670); *Lonicera japonica* (AGE10589); *Angelica gigas* (AEA72280). Accession numbers for (B): *Carthamus tinctorius* (JN998609); *Cynara scolymus* (AM418588); *Chrysanthemum boreale* (KC202425); *Lactuca sativa* (AF299330); *Picrorhiza kurrooa* (JQ996410); *Ipomoea batatas* (D78640); *Melissa officinalis* (FN665700); *Lilium* spp. (AB699156); *Liriodendron tulipifera* (EU190449); *Medicago falcate* (JN849814); *Camellia chekiangoleosa* (JN944578); *Raphanus sativus* (AB087212); *Vaccinium myrtillus* (AY123770); *Cichorium intybus* (EF528572). PAL–HAL family conserved domain in safflower PAL sequence is marked by red line in (A). The bootstrap support values are specified on the nodes. The scale bar indicates 0.2 substitutions per site.

### Conserved domains, homology and phylogenetic analyses of *Ct*CHS

Bioinformatics analysis of *Ct*CHS aa sequence in conserved domain platform confirmed that the isolated region of *Ct*CHS possesses the CHS_like (cd00831) conserved domain [44] including chalcone and stilbene synthases (Figure 3A). As well, a malonyl-CoA binding site delivering the substrate to the active site cysteine [45,46] is detected in safflower CHS. In fact, the members of condensing enzymes superfamily (cl09938), which are capable of catalysing a claisen-like condensation reaction, are engaged in metabolism of fatty acids and biosynthesis of natural products polyketides [47,48] suggesting a similar activity for safflower CHS. From the homology point of view, *Ct*CHS (GenBank: AFI57883) retains considerable identities to its orthologues in *C. chinensis* (96%), *L. sativa*, *S. marianum*, *G. bicolor*, *R. hirta* (95%), *Dahlia pinnata* (94%), *Chrystanthemum nankingense* (93%) and *A. adenophora* (92%). The aa sequences of CHS orthologues in Asteraceae show, as well, a very considerable conservation (Figure 3B), which is rooted from the rather conserved nucleotide sequences of CHS orthologues in this family, forming a distinct branch in corresponding phylogenetic tree (Figure 3B). Likewise, CHS looks highly conserved in members of Brassicaceae family (*Rorippa islandica*, *Cardamine maritime*, *Barbarea vulgaris*, *Arabis setosifolia*, *Brassica oleracea*) making a separate branch (Figure 3B). *Musa acuminata*, *Hypericum hookerianum* and *Zingiber officinale* were as well summoned together in a discrete branch to disclose a more conservation in CHS gene in monocots (Figure 3B). *Ct*CHS partial coding sequence was deposited in GenBank with accession number JQ425086.

**Figure 3:** Amino acid sequence alignment (A) and phylogenetic analysis (B) of CtCHS orthologues Sequence alignment and aa conservation profile for CHS orthologues were generated by ClustalW. Constructions of phylogenetic tree based on nucleotide sequence for CHS gene was carried out by Phylogeny.fr program. Briefly, sequences were aligned with the highest accuracy by MUSCLE. Phylogenetic tree was constructed based upon the maximum likelihood approach executed in PhyML 3.0 software. Graphical demonstration of tree was completed by TreeDyn. Accession numbers for (A): *Carthamus tinctorius* (AFI57883); *Pericallis cruenta* (ACF75870); *Silybum marianum* (AFK65634); *Lactuca sativa* (BAJ10380); *Gynura bicolor* (BAJ17656); *Rudbeckia hirta* (ABN79673); *Dahlia pinnata* (BAK08888); *Ageratina adenophora* (ACQ84148); *Vitis vinifera* (BAA31259); *Litchi chinensis* (ADB44077); *Lilium speciosum* (BAE79201); *Gossypium hirsutum* (ACV72638); *Hypericum hookerianum* (ABM63466). Accession numbers for (B): *Carthamus tinctorius* (JQ425086); *Centaurea jacea* (EF112474); *Rudbeckia hirta* (EF070339); *Musa acuminata* (KF594422); *Acacia confuse* (JN812063); *Rorippa islandica* (DQ399107); *Cardamine maritime* (DQ208973); *Barbarea vulgaris* (AF112108); *Siraitia grosvenorii* (GU980155); *Arabis setosifolia* (JQ919899); *Daucus carota* (AJ006780); *Hordeum vulgare* (EU921436); *Tetracentron sinense* (DQ366573); *Hypericum hookerianum* (EF186910); *Zingiber officinale* (DQ851166); *Brassica oleracea* (AY228486); *Polygonum cuspidatum* (EU647246); *Syzygium malaccense* (GU233757). The conserved domains of chalcone and stilbene synthases are marked by red (Chal-sti-synt-N-terminal) and green (Chal-sti-synt-C-terminal) lines in (A). The bootstrap support values are specified on the nodes. The scale bar indicates 0.5 substitutions per site.

### Effects of SA treatment on *Ct*PAL and *Ct*CHS gene expression profiles

Following treatment of safflower with 0.1 mM SA, as a stimulus of plant responses to pathogen attacks [5], CtPAL transcription levels in different time points were monitored. Accordingly, a slight induction of *Ct*PAL gene was observed at 3-6 hat and levelled off thereafter (Figure 4A). On the other hand, for *Ct*CHS gene only at 3 hat, a noticeable induction was observed (Figure 4A). In contrast, treatment of safflower plants with 1 mM SA had a dramatic influence on both genes expression. Indeed, 1 mM SA treatment led to a biphasic induction pattern of *Ct*PAL gene in 3-6 as well as 24 hat, out of which the latter was much stronger, followed by calming down during the next 24 h (Figure 4B). Concerning *Ct*CHS gene expression after 1 mM SA treatment, a comparable but more augmented expression pattern like that after 0.1 mM SA treatment was observed. A high induction of *Ct*CHS soon after treatment was detectable peaking at 3 hat, followed by a fast decline in expression (Figure 4B). A slight rise in *Ct*CHS expression was also observed at 24 hat.

**Figure 4:** Expression patterns of *Ct*PAL and *Ct*CHS genes after SA treatment with 0.1 mM (A) and 1 mM (B) concentrations Samplings were done at 0, 3, 6, 12, 24 and 48 hat. RNAs were extracted from all seedlings and treated with DNaseI. Subsequently, RNAs were reverse transcribed to corresponding cDNAs. Different PCR products intensities were referred to as temporal expression level of the genes. 18S rRNA transcription levels were considered as internal house-keeping gene control. Sizes of amplicons: *Ct*PAL: 267 bp; *Ct*CHS 559 bp; 18S rRNA: 199 bp.

We treated the safflower plants with two different concentrations of SA, 0.1 and 1 mM, in order to investigate SA-dependency of *Ct*PAL and *Ct*CHS expressions. Seeing that one of the metabolic pathways for SA biosynthesis is succored by PAL activity, the latter stronger induction in PAL transcription might be related to induction of *Ct*PAL by exogenous SA treatment. Generally, plants respond to environmental stresses, e.g. wounding, pathogen attacks, etc. in three main phases [49,50], i.e. (i) development of a physical barrier in the immediate vicinity of wounding or penetrating micro-organism, (ii) activation of defence genes, transiently, neighbouring the stressed site, and (iii) comparatively late systemic activation of defence genes in a rather long-lasting way, of which the first two are almost concomitant. In other word, biphasic induction of gene activation proposes that those distinct phases might be triggered by distinctive signalling incidents; a quick initial induction in response to immediate imposed stress and the slow subsequent response to a generated stress signal [49]. This general pattern is also observed in this study for *Ct*PAL and *Ct*CHS in response to 1 mM SA (Figure 4B). A comparable expression pattern for both PAL and CHS in alfalfa cell suspension culture treated with yeast elicitor was also observed as such the CHS expression maximized at 3 hat and continued with half strength till 24 hat, whereas expression of PAL was transient [51]. Similarly, 1 mM SA treatment caused a biphasic induction of C4H in safflower [4] supporting that expressions of PAL and C4H are coordinated in safflower in response to environmental stresses. As observed in the present study, higher concentration of SA has a more drastic effect on responsiveness of *Ct*PAL and *Ct*CHS than lower concentration. This observation substantiates the crucial role of SA in triggering the phenylpropanoid pathway, which *per se* leads to activation of flavonoid biosynthetic pathway, denoted in induction of respective *Ct*PAL and *Ct*CHS. In fact, elevation of SA level triggers the SAR (systemic acquired resistance), which immunizes the plants towards upcoming pathogen attacks [52].

### Effects of wounding stress on *Ct*PAL and *Ct*CHS gene expression profiles

As phenylpropanoid pathway takes clear task in plant responses to wounding [4,52,53], to characterize the engagement of PAL and CHS in safflower response to wounding, their expression patterns were checked in a 48-h time-frame after leaf injury. Consequently, a slight induction of *Ct*PAL was observed at 3 hat, which lasted in a half strength level till 24 h (Figure 5A). There was no detectable *Ct*PAL expression at 48 h after wounding. In contrast, a much prominent induction of *Ct*CHS in response to wounding was observed especially at 3 hat followed by a gradual decline of transcription till 24 hat (Figure 5A). Similar to *Ct*PAL, no evident expression could be observed for *Ct*CHS at 48 hat. These results suggest that *Ct*CHS, as a key enzyme in flavonoid pathway [26], plays a more critical role in safflower response to wounding than *Ct*PAL. However, in *Scutellaria baicalensis* cell suspension, SbPAL1 gene expression elevated in 1-3 h after wounding and decreased afterward, while SbPAL2, SbPAL3 and SbCHS climaxed at 24 h after wounding [53]. As well, in artichoke, wounding stress led to induction of PAL genes in the first 3 h after stress [24]. As observed by Sadeghi et al. [4], wounding causes the induction of safflower cinnamate 4-hydroxylase (CtC4H) at 3 hat. It appears that the expressions of *Ct*PAL and CtC4H, like their behaviours in response to the SA treatment, are coordinated in safflower in response to wounding similar to coordination of PAL1, 4CL (4-Coumarate:CoA ligase), and C4H in Arabidopsis in response to light and wounding [54]. It is, also, observed that in lettuce induction of PAL gene in response to wounding starts at 6 hat and peaks at 24 hat [55]. Based on our findings, we conclude that in safflower, *Ct*CHS plays a stronger role in wound response than *Ct*PAL. In fact, flavonoid pathway getting started with CHS (Figure 1) is in charge of production of secondary metabolites, which contribute to cell wall fortification as a defence response [4]. Results of this study demonstrate that the phenylpropanoid pathway in safflower, through which lignin biosynthesis occurs, becomes activated soon after injury (Figure 5A) to boost up (i) the biosynthesis of SA as a crucial signalling molecule in plant immunity by induction of *Ct*PAL (this study) and *Ct*C4H [4] and (ii) induction of downstream flavonoid pathway leading to production of phenolic compounds necessary for cell wall fortification by induction of *Ct*CHS.

**Figure 5:** Expression patterns of *Ct*PAL and *Ct*CHS genes after wounding (A) and during salinity stress (B) Samplings were carried out at 0, 3, 6, 12, 24 and 48 hat. RNAs were extracted from all seedlings and treated with DNaseI. Subsequently, RNAs were reverse transcribed to corresponding cDNAs. Different PCR products intensities were referred to as temporal expression level of the genes. 18S rRNA transcription levels were considered as internal house-keeping gene control. Sizes of amplicons: *Ct*PAL: 267 bp; *Ct*CHS 559 bp; 18S rRNA: 199 bp.

### Effects of salinity stress on *Ct*PAL and *Ct*CHS gene expression profiles

To our knowledge, there is minute information available, at molecular level, on involvement of phenylpropanoid pathway in plant responses to salinity. We recently reported the engagement of C4H gene in safflower response to salinity stress [4]. To more scrutinize the key players of safflower in this pathway, we monitored the expression profiles of *Ct*PAL and *Ct*CHS genes in saline condition. Consequently, *Ct*PAL expression got slightly induced at 3 hat and decreased later (Figure 5B). This pattern has also been observed by Gao et al. [56] in cotyledon, hypocotyls, and rootlets of *Jatropha curcas* after treatment with 150 mM sodium chloride; however, the highest induction of PAL was detected in roots. Higher induction of PAL may be a defensive reaction to cellular damages due to high salinity level [56]. In corn inbred lines stressed with salinity, PAL gene expression elevated transiently, similar to the antioxidant genes expression patterns in these plants, suggesting a comparable role for PAL in decreasing the oxidative stress imposed by salinity [57]. For *Ct*CHS, a biphasic strong induction pattern at 3 and 24 h after salinity stress was observed (Figure 5B). As discussed earlier, this biphasic pattern in *Ct*CHS expression might reflect the safflower responses to (i) the immediate salinity and (ii) the later produced stress signal, suggesting that *Ct*CHS takes a considerable task in safflower response to salinity. This probably indicates the real involvement of flavonoid defence pathway in salinity stress condition. We could not find any report on involvement of CHS in plant responses to salinity stress; however, this prominent biphasic induction of *Ct*CHS gene expression clearly substantiates a distinctive role for this gene in safflower tolerance to salinity. This hints at the suitability of *Ct*CHS gene for recruitment in breeding programmes headed for salinity tolerance in other plants. Overall, in this study, we provide molecular evidence for the involvement of *Ct*PAL and *Ct*CHS genes in safflower responses to abiotic stresses. In particular, *Ct*CHS might be considered as a promising candidate for improvement of salinity tolerance in plant breeding programmes.
